# Application of Carbon Nanofiber-Modified Concrete in Industrial Building Design

This article has been retracted.

**DOI:** 10.1155/2023/2587551

**Published:** 2023-01-25

**Authors:** Tianjie Liu

**Affiliations:** College of Civil Engineering and Architectural, Hebei University, Baoding 075000, Hebei, China

## Abstract

In order to explore the influence law and action mechanism of carbon nanofibers on the basic mechanical properties of concrete, the author proposes the mechanical properties and microscopic mechanism of carbon nanofiber-modified concrete. Concrete was prepared with different dosages of carbon nanofibers, and the compressive strength, flexural strength, and splitting strength of carbon nanofiber-modified concrete were tested, and the modification mechanism was explored. Experimental results show that an appropriate amount of carbon nanofibers can improve the mechanical properties of concrete. When the dosage is 0.3%, the mechanical properties of carbon nanofiber-modified concrete are the best, and its compressive strength, flexural strength, and split tensile strength are increased by 9.2%, 13.2%, and 17.5%, respectively, compared with plain concrete. Carbon nanofibers can form a three-dimensional network structure inside the concrete, which can improve the microscopic morphology of the concrete, enhance the toughness and integrity of the concrete, fill the pore defects inside the concrete, refine the pore size distribution, and consume part of the fracture failure energy when the concrete is damaged.

## 1. Introduction

As we all know, the three major building materials widely used in civil engineering are cement, steel, and wood [1]. Concrete is composed of cement and sand aggregates and has compressive strength, as well as resistant to water, fire, and corrosion. In recent years, there has been a lot of research and development in the process of housing planning. It would also be the first choice of people in the home appliance industry in the 20th century. However, because concrete is a hard material with poor tensile strength, reinforced concrete using steel as a supporting material greatly improves the tensile and flexural strengths of concrete. Steel bars are not corrosion-resistant, and in a harsh environment, corrosion is strong and the strength of concrete is lost, so the structure cannot achieve the design model design. In the development of building materials, new problems are constantly arising, and people are constantly seeking new reinforcing materials to replace steel bars. The main research objects are carbon fiber (CFRP), aramid fiber (AFRP), and glass fiber (GFRP) [2]. Carbon fiber has become the focus of research on concrete reinforcement due to its advantages of electrical conductivity, light weight, high strength, large modulus, corrosion resistance, and high temperature resistance.

Carbon fiber is a high-strength, high-modulus, corrosion-resistant, electrically and thermally conductive fibrous carbon material developed in the 1960s [3]. Carbon fiber reinforcement not only improves the flexural and tensile strengths of cement composite materials but also increases the toughness of cement materials, giving traditional cement building materials new properties (light weight, high strength, impact resistance, shrinkage resistance, electrical conductivity, and so on). This makes carbon a very ideal building material. Carbon fiber-reinforced cement concrete (CFRC) is a composite material that was researched and developed in the 1970s. Studies have shown that carbon fiber cement-based composites overcome the shortcomings of cement-based materials such as low tensile strength and flexural strength and large drying shrinkage and have high tensile strength, good impermeability, and a good inhibitory effect on concrete cracks caused by temperature stress, shrinkage, and creep, and the impact resistance and fatigue resistance are greatly improved.

Also, the dispersibility and electrical stability of carbon fiber in cement matrix are still outstanding issues, which directly affect the mechanical properties and pressure sensitivity of carbon fiber cement-based composites. Due to the difficulty in dispersing carbon fiber, the mechanical and electrical properties of its cement base and concrete are not stable enough. Regarding the dispersion of carbon fiber, relevant scholars have done in-depth research, but the problem has not been fundamentally solved. It is still difficult to apply a large number of projects in engineering, and the high price of carbon fiber also limits its wide application. Therefore, we need to seek conductive materials that have good compatibility with cement-based materials, do not affect their mechanical properties, and have good pressure sensitivity. The emergence of nanomaterials makes us see the light of day. Nanocarbon black is one of the cheaper nanomaterials; it has excellent electrical conductivity and high diffusivity, small size, large specific surface area, and excellent interface properties. It can be spread evenly in the cement matrix without dispersant, which not only reduces the artificial strength and high sensitivity of the cementitious and rock pressure-sensitive materials but also improves their stability and makes them less expensive. The sensitivity of nanocarbon black stone materials is good. It is a good business and shows a promising future of use.

## 2. Literature Review

Among the carbon nanofiber-reinforced composite materials, the most studied matrix materials are mainly metal-based, polymer-based, and so on. There are few studies on composite materials with cement-based materials as the matrix, and they are still in their infancy. The research focus mainly includes the dispersion of carbon nanofibers in the matrix and the mechanical properties and durability of carbon nanofiber cement-based composites. Due to the high ratio of carbon nanofibers and strong van der Waals force, carbon nanofibers are prone to agglomeration and entanglement, so it is difficult to achieve a uniform dispersion state in cementitious materials, paper, which cannot improve the effect. In addition, agglomerated carbon nanofibers, like impurities in cement materials, inhibit the hydration of the cement and ultimately affect its microscopic morphology. Foreign researchers have carried out detailed research on the dispersion of carbon nanofibers and carbon nanofiber cement-based composites and often use a combination of ultrasonic treatment and dispersion to uniformly disperse carbon nanofibers in cementitious materials.

Setiawan et al. used a polycarboxylic acid superplasticizer as a dispersant, and with the ultrasonic process, the carbon nanofibers were uniformly dispersed in the aqueous solution. The dosages of 0.1% and 0.2%, respectively, were applied to the cement-based materials, and the water-cement ratio was 0.4. The mechanical properties of carbon nanofiber cement-based composites were studied at 7 days, 14 days, and 28 days, respectively, including flexural strength, fracture deformation, ultimate strain, and toughness. The dispersion of carbon nanofibers in the matrix is also discussed. The results of the study showed that at 7 and 14 days of age, carbon nanofibers had no obvious enhancement effect on cement-based materials, but at 28 days, the mechanical properties (fracture deformation, flexural strength, ultimate strain, and toughness) of carbon nanofiber cement-based composites were all higher than those of blank samples [4]. Abregú et al. used polycytic acid superplasticizer as dispersant and firstly prepared carbon nanofiber dispersion suspension by the ultrasonic method. Then, the prepared suspension is applied to cement concrete to prepare nanocarbon fiber cement-based composite material [5]. The results show that the dispersion state of carbon nanofibers is regional. The carbon nanofibers are not uniformly dispersed on the fracture surface, so the dispersion effect is not very good. At the same time, the relationship between the particle size of cement and the dispersion of carbon nanofibers was discussed. When a large amount of carbon nanofibers is added, the larger the cement particles are, the more unfavorable their dispersion is in the cement matrix. Rajeshwari et al. applied silica fume to carbon nanofiber cement-based composites, and the content of carbon nanofibers was 2 wt%. The research results show that the addition of silica fume is beneficial to the dispersion effect of carbon nanofibers in the cement-based matrix. The bonding strength of carbon nanofibers to a cement-based matrix is also enhanced. At the same time, the addition of carbon nanofibers can effectively improve the pore structure of the composite material, make the body more compact, and cause the pores change to a smaller size [6]. Maleki et al. studied the mechanical properties of carbon nanofiber cement-based composites, and the content of carbon nanofibers was 0.048 wt%. In order to improve the dispersibility of carbon nanofibers in the cement-based matrix, dispersant and ultrasonic treatment were firstly applied to prepare a uniformly dispersed aqueous solution of carbon nanofibers. When the ultrasonic capacity is 2800 kJ/1 and the ratio of dispersant to carbon nanofibers is 4 : 1, the best dispersion suspension can be obtained [7].

The author intends to prepare nanocarbon fiber reinforced cement concrete specimens, starting from the strength indicators such as compressive strength, flexural strength, and splitting strength, and explore the influence law and mechanism of carbon nanofibers on the basic mechanical properties of concrete; the modification effect of carbon nanofibers on concrete is explored from the microscopic level in order to provide a theoretical basis and application basis for the research and application of high-durability protective materials and to make up for the deficiencies in the existing research on carbon nanofiber modified concrete.

## 3. Research Methods

### 3.1. Test

#### 3.1.1. Preparation of Raw Materials and Test Pieces

The raw materials used are cement: P·O 42.5R grade cement; sand: medium sand with a fineness modulus of 2.9, an apparent density of 2620 kg/m^3^, and a mud content of 1.1%; limestone crushed stone: large crushed stone (apparent density 2730 kg/m^3^) and small crushed stone (apparent density 2644 kg/m^3^) are mixed in a mass ratio of 7 : 3; water reducing agent: polycarboxylate high-performance water reducing agent (see Table 1 for performance); defoaming agent: tributyl phosphate defoaming agent, content 99.6% and density of 0.974∼0.980 g/cm^3^; fiber: carbon nanofiber (see Table 2 for technical parameters).

A total of two types of specimens were prepared for the test: a cube specimen of 100 mm × 100 mm × 100 mm and a prismatic specimen of 100 mm × 100 mm × 400 mm [8, 9]. The preparation steps are as follows: ① preparation of carbon nanofiber dispersion: mix the water reducing agent into the water and stir evenly, add carbon nanofibers and half-part defoamer, stir at high speed for 2 minutes, add the remaining half-part defoamer, and manually stir at low speed for 5 minutes until there are no obvious bubbles in the dispersion; ② preparation of the concrete mixture: mix cement, sand, and stone evenly by the dry mixing method, then add nanocarbon fiber dispersion while stirring, and finally stir for 2 minutes; and ③ pouring and curing: after pouring and forming, cure under standard conditions for 28 d. The test mix ratios are shown in Table 3.

### 3.2. Test Method

In accordance with the methods in GB 50081-2002, “Standards for Mechanical Properties of Ordinary Concrete,” the basic mechanical properties of concrete specimens were tested. Among them, the compressive strength test uses an electrohydraulic servo compressive testing machine to pressurize the cube specimen; when the specimen is close to failure, stop adjusting the throttle until it breaks, record its load-displacement curve, and multiply the test result by a conversion factor of 0.95. The flexural strength test uses a flexural testing machine to test the prismatic specimen [10]. The test result needs to be multiplied by a conversion factor of 0.85. The splitting strength test uses the electrohydraulic servo test system and the split-pull test device to conduct the split-pull test on the cube specimen, and the test results need to be multiplied by the conversion factor of 0.85.

## 4. Analysis of Results

### 4.1. Compressive Strength

Figure 1 is a graph showing the effect of carbon nanofiber content on the compressive strength of concrete. It can be seen from Figure 1 that ① when the content of carbon nanofibers is 0.1%, 0.2%, 0.3%, and 0.4%, the compressive strength of concrete is increased by 2.5%, 6.1%, 9.2%, and 6.8%, respectively; compared with ordinary concrete, it shows that an appropriate amount of carbon nanofibers can effectively improve the compressive strength of concrete, and the improvement effect is the best when the dosage is 0.3%; ② when the content of carbon nanofibers is 0.5%, the compressive strength is reduced by 1% compared with ordinary concrete; and ③ with the increase of the content of carbon nanofibers, the compressive strength of concrete increases first and then decreases, indicating that carbon nanofibers cannot be added to the concrete blindly; too much carbon nanofibers will not only reduce the improvement effect but also cause waste of resources [11]. The following is the formula for calculating the compressive strength:

(1) $$\begin{array}{c} f_{cu}=\frac{F_{\max}}{A}\text{.} \end{array}$$

In the formula, *f*_*cu*_ is the compressive strength of concrete cube (MPa); *F*_max_ is the maximum load (N); and *A* is the cross-sectional area of specimen under compression (mm^2^).

### 4.2. Flexural Strength

Figure 2 shows the effect of carbon nanofiber content on the flexural strength of concrete. It can be seen from Figure 2 that ① when the content of carbon nanofibers is less than 0.3%, the flexural strength of carbon nanofiber-reinforced cement concrete increases with the increase of the content. After the dosage exceeds 0.3%, the flexural strength of concrete decreases sharply with the increase of the dosage [12]. When the content of carbon nanofibers is 0.1%, 0.2%, 0.3%, and 0.4%, the flexural strength of carbon nanofiber-reinforced cement concrete is increased by 3.7%, 8.9%, 13.2%, and 7.3%, respectively, compared with ordinary concrete. The improvement effect is the best when the amount is 0.3%; ② when the dosage is 0.5%, the flexural strength of carbon nanofiber-reinforced cement concrete is 5.2% lower than that of ordinary concrete, indicating that adding too much carbon nanofibers will not only not improve the flexural strength of concrete but even deteriorate its flexural strength [13, 14].

### 4.3. Split Tensile Strength

Figure 3 shows the effect of carbon nanofiber content on the splitting tensile strength of concrete. It can be seen from Figure 3 that ① when the content of nanocarbon fiber is less than 0.3%, with the increase of the content, the splitting tensile strength of nanocarbon fiber-reinforced cement concrete increases continuously, but when the content exceeds 0.3%, the splitting tensile strength decreases sharply [15]. When the content of carbon nanofibers is 0.1%, 0.2%, 0.3%, and 0.4%, the splitting tensile strength of carbon nanofiber-reinforced cement concrete is increased by 2.8%, 10.8%, 17.5%, and 9.5%, respectively, compared with ordinary concrete. The improvement effect is more obvious when the amount is 0.2%∼0.3%; ② when the amount is 0.5%, the split tensile strength of carbon nanofiber-reinforced cement concrete is 6.3% lower than that of plain concrete, indicating that the increase of carbon nanofibers deteriorates the tensile strength of concrete [16].

### 4.4. Modification Mechanism

#### 4.4.1. Distribution of Carbon Nanofibers in Concrete

There are a lot of holes in ordinary concrete, the hydration products are in a loose state, and the integrity is poor. When the dosage is 0.1%, the carbon nanofibers are sparsely distributed in the concrete, and only a few sporadically interspersed in the gel material can be seen under the scanning electron microscope, so the modification of concrete is of little significance. Continuing to increase the dosage, the carbon nanofibers are distributed more and more widely in the concrete, and the hydration products are interwoven vertically and horizontally, overlapping each other into a three-dimensional network structure, and the material integrity is gradually strengthened. The crystal form of the hydration product is smaller than that of ordinary concrete, and when the dosage is 0.3%, the distribution and modification effect of carbon nanofibers in concrete are better [17]. Carbon nanofiber particles have high surface activity, which can accelerate the hydration of cement when incorporated into concrete. Due to the nucleation and adsorption of nanomaterials, the hydration product gradually forms a network structure with nanoparticles as the core, which inhibits the formation of large crystals and reduces the degree of crystal orientation; thereby, the interface structure between cement stone and aggregate is improved, and the strength of concrete is improved. When the dosage is 0.4%, the strong van der Waals force makes carbon nanofibers agglomerate in a small area. When the dosage is 0.5%, the agglomeration phenomenon is more obvious, the distribution of carbon nanofibers in the hydration products around the agglomerates is significantly reduced, and the carbon nanofibers are difficult to play their modification role. It will even cause a weak area inside the concrete, resulting in a concrete strength lower than that of plain concrete without carbon nanofibers, which will adversely affect the mechanical properties and durability of the concrete [18].

### 4.5. Molecular Chain Effect of Carbon Nanofibers

Carbon nanofiber monofilaments are wrapped by C-S-H gel particles, which connect the gel particles together like molecular chains, thereby enhancing the toughness and integrity of the gel.

### 4.6. Filling Effect of Carbon Nanofibers

Carbon nanofibers are very small in size and can have a small size effect when mixed into concrete, filling part of the pore defects of the concrete, effectively reducing the content of macropores in concrete and improving the particle gradation of cementitious materials. The fine pores are filled in the structure, the pore structure is refined inside the concrete, and the strength, compactness, and impermeability of the concrete are improved [19].

### 4.7. Bridging Effect of Carbon Nanofibers and Pull-Out and Fracture Effects When Concrete Is Damaged

The fibrous structure of carbon nanofibers bridges the micropores and microcracks inside the concrete structure, effectively preventing the further development of microcracks. At the same time, the molecular chain effect of carbon nanofibers strengthens the connection between the components, enhances the integrity of the concrete, and then improves the strength of the concrete. With the continuous destruction of concrete under the external action, the microcracks gradually expand, and the tensile stress received by the carbon nanofibers in the process of crack development gradually increases and finally pulls out of the cement slurry or directly breaks [20]. In the process of pulling out and breaking, when the carbon nanofibers break free from the bondage of the cement slurry or destroy themselves, part of the breaking energy is consumed, thereby inhibiting the development of microcracks in concrete.

## 5. Conclusion

1. Adding an appropriate amount of carbon nanofibers can improve the mechanical properties of concrete. When the dosage is 0.3%, the basic mechanical strength indicators of the material are the best, and the compressive strength, flexural strength, and split tensile strength are better than those of plain concrete; they are improved by 9.2%, 13.2%, and 17.5%, respectively.
2. An appropriate amount of carbon nanofibers is well dispersed in concrete, which can form a three-dimensional network structure and reduce the crystal form of hydration products.
3. The carbon nanofibers in the modified concrete connect the gel particles together like molecular chains, which enhances the toughness and integrity of the gel.
4. The size of carbon nanofibers is extremely small, which can fill the pore defects in concrete to a certain extent.
5. The carbon nanofibers are bridged between the microcracks of the modified concrete, which can consume part of the fracture failure energy when the concrete is damaged.

## Figures and Tables

**Figure 1:** Compressive strength.

**Figure 2:** Flexural strength.

**Figure 3:** Split tensile strength.

**Table 1:** Performance index of polycarboxylate superplasticizer.

Water reduction rate (%)	Bleeding rate (%)	Gas content (%)	Coagulation time (min)		Compressive strength ratio		Shrinkage ratio (%)
			Initial setting	Final coagulation	3 d	7 d	
≥26	≤65	≤3.5	−65	90	≥150	≥140	≤105

**Table 2:** Technical parameters of carbon nanofibers.

Diameter (nm)	Length (*μ*m)	Resistivity (Ω·cm)	Thermal conductivity [W/(m·°C)]	Specific surface area (m^2^/g)	Thermal expansion coefficient (1/°C)	Bulk density (g/cm^3^)	True density (g/cm^3^)
150∼200	10∼20	<0.012	2000	300	1	0.18	2

**Table 3:** Mixing ratio of test pieces kg/m^3^.

Numbering	Cement	Water	Sand	Gravel	Carbon nanofiber	Water reducer	Defoamer
PC	495	180	672	1008	0	5	3
CNFC01	495	180	672	1008	0.18	7.5	4.5
CNFC02	495	180	672	1008	0.37	10	6
CNFC03	495	180	672	1008	0.55	12.5	7.5
CNFC04	495	180	672	1008	0.71	15	9
CNFC05	495	180	672	1008	0.9	5	3

## Data Availability

The data used to support the findings of this study are available from the corresponding author upon request.
